This article has been retracted.

# CT, MRI, and ^18^F-FDG PET/CT imaging features of seven cases of adult pancreatoblastoma

**DOI:** 10.1186/s12880-022-00958-4

**Published:** 2022-12-29

**Authors:** Mengnan Wu, Jiongbin Lin, Zhuangsheng Liu, Zhiming Huang, Ruoning Wang

**Affiliations:** 1 Department of Radiology, Heyuan People’s Hospital, General Hospital Guangdong, Heyuan, 517000 China; 2 Department of Radiology, Nanfang Hospital, Southern Medical University, Guangzhou, 510515 China; 3 Department of Radiology, The Sixth Affiliated Hospital, South China University of Technology, Nanhai People’s Hospital, Foshan, 528200 Guangdong China; 4 Minimally Invasive Centre, Tumour Hospital, Sun Yat-Sen University, Guangzhou, 510060 China

**Keywords:** Pancreatoblastoma, CT, MRI, PET/CT

## Abstract

**Objective:**

This study mainly analysed the imaging data for seven cases of adult pancreatoblastoma (PB) and summarized additional imaging features of this disease based on a literature review, aiming to improve the understanding and diagnosis rate of this disease.

**Materials and methods:**

The imaging data for seven adult patients pathologically diagnosed with adult PB were retrospectively analysed. Among the seven patients, six underwent computed tomography (CT) scans, two patients underwent abdominal magnetic resonance imaging (MRI), and five patients underwent ^18^F-FDG PET/CT.

**Results:**

The tumours were located in the head of the pancreas in three cases, in the tail of the pancreas in two cases, and in the gastric antrum and neck of the pancreas in one case. Six tumours showed blurred edges, and an incomplete envelope was observed in only two cases when enhanced, which showed extruded growth and cyst-solid masses; one tumour was a solid mass with ossification. Showing mild or significant enhancement in the arterial phase (AP) for six cases. In the MRI sequence, isointensity was found on suppressed T1-weighted imaging, and hyperintensity was noted on suppressed T2-weighted imaging in two cases, with significant enhancement. Pancreatic duct dilatation was found in four cases. Tumour ^18^F-FDG PET/CT imaging exhibited high uptake in five cases.

**Conclusion:**

Adult PB involves a single tumour and commonly manifests as cystic-solid masses with blurred edges. Capsules are rare, ossification is an important feature, tumours can also present in ectopic pancreatic tissues, with mild or strengthening in the AP, and ^18^F-FDG uptake is high. These features are relatively specific characteristics in adult PB.

## Introduction

Pancreatoblastoma (PB) is a rare malignant embryonic tumour of the pancreas with multicellular differentiation [1–3]. Although PB can occur at any age, it occurs mostly in children and rarely in adults. Fewer than 50 cases have been reported since Palosaari et al. reported the first case of adult PB [4–6], and these studies describe only the clinical manifestations and pathological features of adult PB. Surgical resection is the mainstay of treatment, and complete resection has been associated with long-term survival [7]. As the neoplasm consists of multiple cell lines, squamoid corpuscles are distinctive pathological features of PB, and fine needle aspiration or cytology alone is not sufficient; therefore, the imaging techniques are particularly important and useful in diagnosing and staging adult PB.

The purpose of our study was to comprehensively describe the Imaging features of adult PB on computed tomography (CT), magnetic resonance imaging (MRI), and 18F-FDG PET/CT and to provide a literature review.

## Materials and methods

### Clinical data

Imaging data for seven adult patients pathologically diagnosed with PB from November 2012 to April 2021 were retrospectively identified. We collected seven cases from Heyuan People’s Hospital and Nanfang Hospital, Southern Medical University. The patients involved were aged from 26 to 69 years, with an average age of 56 years. This retrospective study was approved by the Ethics Committee of Heyuan People’s Hospital and Nanfang Hospital, and informed consent was not required The clinical manifestations are shown in Table 1.

**Table 1:** Clinical manifestations of adult PB

Case	Age	Sex	Symptom	Genetic syndrome	AFP (0–10 ng/mg)	CA199 (0–27 U/ml)	Follow-up (months)
1	26	F	Abdominal pain	No	/	210.67	NR
2	47	F	Abdominal pain	No	1.90	26.03	NED 24
3	64	F	Change in bowel habits	No	/	35.02	NED 26
4	68	M	Diarrhoea, black stool	No	3.20	40.05	NED 4
5	69	F	Abdominal pain	No	2.50	0.36	NED 4
6	65	F	Abdominal pain and chronic pancreatitis	No	1.30	2.95	NR
7	58	M	Abdominal pain	No	183.3	11.02	NR

### Imaging technique

Six patients underwent noncontrast and contrast-enhanced CT, as shown in Table 2.

**Table 2:** Parameters of CT

Equipment	Period image	Contrast agent	Injection rate	Tube voltage	Tube current	Reconstruction matrix	Reconstruction slice thickness
SOMATOM definition 64/GE revolution/GE optima CT660	AP; PVP; DP	Ioversol injection	3 ml/s	120–130 kV	200–300 mAs	512 × 512	1–1.25 mm

Two patients underwent abdominal MRI, as shown in Table 3.

**Table 3:** Sequences and parameters of Gd-DTPA-dynamic enhanced MRI

Sequences	Image plane	TR/TE (msec)	FOV (mm)	Flip angle	Thickness (mm)	Matrix
FIESTA	BH C	3.6/1.5	400*400	65	5	192*224
T1WI (in-phase /opposed-phase)	BH A	200/4.8(2)	420*420	80	6	288*192
T2WI	A	8576/85	400*400	160	6	320*224
DWI	A	6667/73	420*420	180	5	128*128
LAVA	A	4.0/2.0	420*420	14	2.5	320*288
LAVA	C	4.0/2.0	420*420	14	2.5	320*288

Five examinations were carried out using a GE Discovery LS PET/CT scanner (GE Healthcare, Waukesha, Wisconsin, USA). ^18^F-FDG with a radiochemical purity greater than 95% was obtained using a tracer synthesis system (TRACERlab FXFDG; GE Healthcare, USA). Approximately 60 min after intravenous injection of 318–524 MBq (8.6–14.2 mCi, 150 μCi/kg) of ^18^F-FDG, whole-body PET/CT was performed using 120 kV, 80–250 mA, 0.5-s rotation time, 3.6 pitch, 5-mm slice thickness, and a 512 × 512 matrix without contrast enhancement from the mid-thigh to the head. The acquired CT and PET images were sent to an Xeleris workstation (GE Healthcare). Lesions with increased uptake of 18F-FDG were considered positive tumours.

### Image analysis

The CT and MRI images were evaluated by two radiologists (with 10 and 15 years of experience in abdominal radiology) who were blinded to patient information. Disagreements were resolved by consensus. The focuses of observation and analysis included tumour location, size, morphology, margin, capsule, growth pattern, internal components, contrast-enhanced scanning mode, the presence or absence of lymph node metastasis, adjacent blood vessels, and organ invasion and metastasis.

^18^F-FDG PET/CT was used to analyse the uptake of the lesion (a lesion with uptake higher than that of the adjacent tissues was considered positive), and the brightness (indicating the uptake level) of the solid portion and necrotic area of the tumour was compared. The region of interest was drawn along the margin of the lesion on the PET image, and the standardized uptake value (SUVmax) was measured.

### Pathology

All specimens in this study were reviewed by two pathologists with 10 years of experience to confirm the diagnosis of PB and the presence or absence of tumour necrosis, a capsule, lymph node metastasis, and vascular tumour thrombus.

## Results

### Features of the imaging

The tumours were cyst-solid masses in five cases, and one was a solid mass, located in the head of the pancreas in three cases; two tumours were in the tail of the pancreas, one case was in the gastric antrum, and one case was in the neck of the pancreas (Fig. 1a–c). Six tumours showed blurred edges, and an incomplete envelope noted in only two cases when enhanced (Fig. 2a). One case displayed ossification. Mild enhancement in the arterial phase (AP) was observed in two cases (Fig. 2b), and strengthened enhancement in the AP was observed in four cases (Fig. 2c). Pancreatic duct dilatation was found in four cases. In the MRI sequence, isointensity was found on suppressed T1-weighted (T1WI), and hyperintensity was found on T2-weighted suppressed (T2WI) in two cases (Fig. 3a–b), with significant enhancement (Fig. 3c). ^18^F-FDG PET/CT had a high uptake (Fig. 4a–c) in five tumours.

**Fig. 1:** **a** Data from a 64-year-old female patient with a change in bowel habits lasting 8 months. The tumour was quasi-round, located in the head of the pancreas, showed restricted, bifurcated, and extruded growth, and displayed ossification on noncontrast CT scans, with a CT value of approximately 278.4 HU. **b** Data from a 65-year-old female patient with abdominal pain and chronic pancreatitis lasting 11 months. The pancreas was enlarged, and the tumour was indistinct on noncontrast CT scans. **c** Data from a 68-year-old male patient with diarrhoea and black stool. The tumour was located in the gastric antrum, was quasi-round and cystic-solid, and showed restricted, bifurcated, and extruded growth on noncontrast CT scans

**Fig. 2:** **a** Data from a 26-year-old female patient with abdominal pain. The tumour exhibited an incomplete capsule during the AP (red arrow) on enhanced CT scans. **b** The gastric antrum tumours were mildly enhanced in the AP and not enhanced for necrosis and cysts in the centre on enhanced CT scans. **c** The tumour was significantly enhanced in the AP and not enhanced for necrosis and cysts in the centre on enhanced CT scans

**Fig. 3:** **a**, **b** The tumour appeared isointense on T1WI and hyperintense on T2WI.** c** The tumour was indistinct with significant enhancement in the AP

**Fig. 4:** **a-c** PET/CT showed intense uptake of fluorine-18 fluorodeoxyglucose in the neck of the tumour and liver metastases (red arrow and black arrow)

Details are shown in Tables 4, 5, and 6.

**Table 4:** Imaging features for CT in six patients

Case	1	2	3	4	5	6	7
Location	Head	Head	Head	Antrum of stomach	Tail	Neck	Tail
Size (cm)	4.4 × 6.6	5.8 × 6.4	3.7 × 2.7	4.6 × 3.2	6.4 × 5.3	6.2 × 4.0	3.5 × 2.8
Shape	Round	Round	Round	Round	Irregular	Round	Round
Growth pattern	Localized outgrowth	Localized outgrowth	Localized outgrowth	Localized outgrowth	Localized outgrowth	Diffuse growth	Localized outgrowth
Density	Iso	Iso	Iso	Iso	Iso	Iso	/
Cystic or necrotic component	Yes	Yes	No	Yes	Yes	Yes	**/**
Calcification or Ossification	Calcification	**/**	Ossification	**/**	**/**	**/**	**/**
Margin	Indistinct	Indistinct	Indistinct	Indistinct	Indistinct	Indistinct	/
Capsule	Yes	Yes	No	No	No	No	/
Enhancement	Fast-in and slow-out	Fast-in and slow-out	Fast-in and slow-out	Slow-in and slow-out	Slow-in and slow-out	Fast-in and slow-out	**/**
Pancreatic duct obstruction	Yes	Yes	Yes	No	No	Yes	/

**Table 5:** MRI features in two patients

Case	1	2	3	4	5	6	7
T1WI	/	/	/	Iso	/	Iso	/
T2WI	/	/	/	Hyper	/	Hyper	/
DWI	/	/	/	Hyper	/	Hyper	/
Margin	/	/	/	Sharp	/	Indistinct	/
Enhancement	/	/	/	Fast-in and slow-out	/	Fast-in and slow-out	/

**Table 6:** 18F-FDG PET/CT features in five patients

Case	1	2	3	4	5	6	7
^18^F-FDG PET/CT	Uptake	Uptake	/	/	Uptake	Uptake	Uptake
SUVmax	13.2	6.5	/	/	10.3	11.2	11.6
Metastasis	Liver	No	No	Lymph node	Kidneys adrenal	Liver pancreas	Liver lymph node

### Details of the pathology

In general, the tumour boundaries were well defined (Fig. 5a). Six tumours were greyish-white in the periphery and light yellow at the centre, and one tumour was light yellow. Microscopic examination revealed that all tumour tissues were acinar-like and duct-like with squamous corpuscles (Fig. 5b). Immature bone was visible in tumour cells in one case (Fig. 5c), and tumour cells were rich in interstitial fibroblasts in two cases. Immunohistochemical staining of acinar differentiation markers mainly included trypsin and chymotrypsin, and neuroendocrine markers mainly included CD56, CgA, Syn, and α-AT.

**Fig. 5:** **a** In general, the tumour was light yellow. **b** HE staining (20 × 20) showed squamous corpuscles (black arrow). **c** Ossification was visible in tumour cells

## Discussion

Adult PB is a rare exocrine pancreatic malignancy, and the clinical manifestations are diverse and nonspecific. At present, the literature mainly focuses on case reports. Because of a lack of familiarity with this disease among clinicians and radiologists, the diagnosis is often inaccurate or delayed. Adult PB is usually misdiagnosed as other tumours by CT and/or MRI scans, However, the final diagnosis mainly depends on histopathological tests, but through multimodal imaging technology, with retrospective reanalysis and reevaluation of our study and in combination with supporting research, we found several imaging features indicating and/or supporting the diagnosis of adult PB.

PB is a single mass, shown as a cyst-solid or solid mass, with cyst-solid being more common [8–10]. Corrias [5] found that most tumours are located in the head of the pancreas, and pancreas head tumours accounted for 43% of our cases. We support the head of the pancreas as the most common site. Ectopic pancreatic PB has not been reported in previous literature, and we found that it can occur in the gastric antrum in our study. These tumours were isodense on CT scans with low density in the centre and had sandy calcifications and ossification, which is consistent with PB consisting of multiple cell lines [11, 12]. No pathology or imaging has been reported for ossification. We considered that pancreas tumours with ossification are evident on CT, and the possibility of adult PB should be considered, which is an important feature. PB was well circumscribed with a good capsule, and dilation of the pancreatic duct was rare [13, 14]. In contrast to previous literature reports, we found that the edges of the masses were blurred, and an incomplete envelope was shown in only two cases when enhanced in our study, which is possibly related to PB having highly aggressive growth [15]. Pancreatic duct dilatation was found in our study, with tumour tissue in the pancreatic duct observed on microscopic examination, which indicates that pancreatic duct dilation caused by adult PB is common. Mild enhancement was observed in enhanced scans in a previous report [9]. Mild enhancement in the AP was observed in two tumours in our study, showing a slow-in and slow-out pattern, similar to previous reports. In contrast to the literature reports, four cases had strengthened enhancement in the AP, showing a fast-in and slow-out pattern. The strengthened enhancement is related to the pathology finding of a vascular structure around the squamoid corpuscles, which is a new finding that will be helpful for diagnosing adult PB. In the MRI sequence, isointensity was found on T1WI, while hyperintensity was found on T2WI in two cases, with limited diffusion [9]. Contrast-enhanced scans were consistent with CT scans, with significant enhancement in the AP [1, 16]. MRI can more clearly show the malignant behaviour of adult PB and is helpful for clinicians to presurgically assess whether the tumour can be completely removed. With metastases at different sites, mainly including the liver followed by the lymph nodes [15, 17], as in our study, a pancreatic tail lesion may invade the left kidney, which is in agreement with reports that PB is prone to invade adjacent structures.

The reviewed papers revealed [9] that the tumour does not exhibit FDG uptake on 18^F−^FDG PET/CT examination. In our study, ^18^F-FDG PET/CT had high uptake in five tumours. The SUV_max_ average value was 10.56. One of the patients had pancreatitis, pancreas enlargement, an indistinct tumour on CT and MRI, and clear, high uptake on ^18^F-FDG PET/CT. Zhou et al. [18] found that ^18^F-FDG and ^68^ Ga-DOTATATE PET/MR were acquired for presurgical assessment of adult PB invasion and malignant potential, which revealed intense FDG uptake and mild DOTATATE uptake. We believe that ^18^F-FDG PET/CT is an imaging modality for sensitive detection of pancreatic malignancies.

Adult PB and pancreatic cell tumours share many clinical and morphological similarities, and distinguishing between them is difficult. Thus, definitive diagnosis of PB depends on pathological examination characterized by the presence of squamous cell nests with prominent acinar differentiation and foci of ductal, squamous, and endocrine cells [19, 20].

*Limitations* Because adult PB is extremely rare, this retrospective study had a small sample size. Our findings should be confirmed by further studies with large samples.

*Follow-up* Adults with PB have a worse prognosis than children with PB at 20 months following chemoradiotherapy and surgery [20]. The longest survival time among our patients was 26 months.

In conclusion, adult PB involves a single tumour and commonly manifests as cystic-solid masses with blurred edges. Capsules are rare, ossification is an important feature, tumours can also present in ectopic pancreatic tissues, with mild or strengthening in the AP, and ^18^F-FDG uptake is high. Combining contrast CT and MRI, 18F-FDG PET/CT is the best choice for accurate diagnosis preoperatively, which is critical for directing future treatment.

## Data Availability

The raw data may be made available upon reasonable request from the corresponding author.

## Abbreviations

NR: Not reported
NED: No evidence of disease
A: Axial
C: Coronal
BH: Breath hold
Iso: Isodense/isointense
Hyper: Hyperintense
